# Salvage Liver Transplantation for Patients with Recurrent Hepatocellular Carcinoma after Curative Resection

**DOI:** 10.1371/journal.pone.0041820

**Published:** 2012-07-26

**Authors:** LinWei Wu, AnBin Hu, Ngalei Tam, JianWei Zhang, Min Lin, ZhiYong Guo, XiaoShun He

**Affiliations:** 1 Organ Transplant Center of the First Affiliated Hospital, Sun Yat-sen University, Guangzhou, China; 2 Zhongshan Medical School of Sun Yat-sen University, Guangzhou, China; University of Colorado, United States of America

## Abstract

**Objective:**

To summarize the experience with salvage liver transplantation (SLT) for patients with recurrent hepatocellular carcinoma (HCC) after primary hepatic resection in a single center.

**Methods:**

A total of 376 adult patients with HCC underwent orthotopic liver transplantation (OLT) at Organ Transplantation Center, the First Affiliated Hospital of Sun Yat-sen University, between 2004 and 2008. Among these patients, 36 underwent SLT after primary liver curative resection due to intrahepatic recurrence. During the same period, one hundred and forty-seven patients with HCC within Milan criteria underwent primary OLT (PLTW group), the intra-operative and post-operative parameters were compared between these two groups. Furthermore, we compared tumor recurrence and patient survival of patients with SLT to 156 patients with HCC beyond Milan criteria (PLTB group). Cox Hazard regression was made to identify the risk factors for tumor recurrence.

**Results:**

The median interval between initial liver resection and SLT was 35 months (1–63 months). The intraoperative blood loss (*P*<0.05) and transfusion volume (*P*<0.05) were larger in the SLT group than in the PLTW group. The operation time was longer in the SLT group (*P*<0.05). The post-operative complications incidence, tumor recurrence rate, patients' survival rate, and tumor-free survival rate were comparable between these two groups (all *P*>0.05). When compared to those patients with HCC beyond Milan criteria undergoing primary OLT, patients undergoing SLT achieved a better survival and a lower tumor recurrence. Cox Proportional Hazards model showed that vascular invasion, including macrovascular and microvascular invasion, as well as AFP level >400 IU/L were risk factors for tumor recurrence after LT.

**Conclusions:**

In comparison with primary OLT, although SLT is associated with increased operation difficulties, it provides a good option for patients with HCC recurrence after curative resection.

## Introduction

In China mainland, the incidence of hepatocellular carcinoma (HCC) is increasing, and it is the third leading cause of cancer mortality [1]. Orthotopic liver transplantation (OLT) remains the most effective treatment for patients with small HCC. However, due to organ shortage, economic or conceptional constraints, only a small population of such patients could receive a transplant. Hepatic resection (HR) remains a more reasonable choice for the vast majority of such patients although they might face a higher risk of tumor recurrence or liver function deterioration. However, for those patients with HCC recurrence after hepatic resection, 80% might be rescued by means of liver transplant [2], [3]. The concept of liver transplant performed after HCC recurrence post HR, namely salvage liver transplantation (SLT) has been introduced by Pietro E. Majno [2] in 2000. Herein we retrospectively reviewed and compared the patient survival and cancer recurrence rates between patients undergoing SLT and primary OLT in our single center between 2004 and 2008.

## Methods

### Baseline characteristics of patients

From January 2004 to December 2008, 376 adult patients with HCC received OLT at our center, including 296 males and 80 females (mean age, 50.8 years; age range, 18–75 years). The patients who had tumor thrombosis of the main trunk of portal vein or hepatic vein (vena cava) (n = 19), and those who had ABO incompatible match (n = 8), had split grafts (n = 6) and living donors (n = 4) were excluded from this study.

Thirty-six patients received SLT after radical HR due to intra-hepatic recurrence. All the 36 patients were included in the SLT group. One hundred and forty-seven patients who received primary OLT for HCC within Milan criteria were classified into PLTW (primary OLT for HCC within Milan criteria) group. The demographics and clinical data of the patients in the two groups are shown in Table 1. There was no significant difference in pre-operative baseline characteristics between the two groups. We also compared the tumor recurrence and patients survival of SLT group to 156 patients undergoing primary OLT for HCC beyond Milan criteria (PLTB group), and the risk factors for tumor recurrence was identified by Cox regression analysis.

**Table 1:** Demographics of the patients.

	SLT (*n* = 36)	PLTW (*n* = 147)	PLTB (n = 156)	*P* value
Age (yr)				
Mean ± SD	49.4±17.1	47.6±15.8	51.1±15.6	0.160
Median	48 (20–65)	49 (18–63)	46(22–68)	
Gender(M/F)	27/9	106/31	118/38	0.775
HBV infection	35 (97.2)	144 (97.9)	149(95.5)	0.479
HCV infection	2 (5.5)	9 (6.1)	11(7.1)	0.921
ALT (IU/L)	110.5±90.2	100.4±84.8	122.7±88.6	0.085
Sodium (mmol/L)	137.9±7.3	139.4±6.8	141.1±9.8	0.059
Albumin (mg/L)	36.9±17.9	38.8±20.9	34.9±21.5	0.269
Creatinine (µmol/L)	95.5±93.2	86.8±95.3	105.1±89.8	0.229
Bilirubin(µmol/L)	48.3±39.6	57.2±46.5	60.5±37.3	0.282
INR	1.59±0.48	1.60±0.59	1.75±0.62	0.065
MELD score	18.6±6.7	17.9±7.1	19.4±4.8	0.103
Liver cirrhosis	36(100%)	131(89.1%)	104(66.7%)	<0.001
Tumor demographics				
Nodules numbers				
solitary	21	86	40	<0.001
≤3	13	61	56	0.580
>3	2	0	60	<0.001
Largest tumor size(mm)	48	50	130	0.465
AFP levels (IU/L)				
<400	12	44	10	<0.001
≥400	24	103	146	<0.001
Macro vascular invasion	0	0	37	<0.001
Microvascular invasion	2	14	55	<0.001
Pathologic characteristics				
Poor differentiated	8	30	68	<0.001
Well differentiated	28	117	88	<0.001
Pre-transplant treatment				
radiofrequency ablation	9	34	25	0.224
ethanol injection	6	25	30	0.860
TACE	3	14	18	0.777

Abbreviation: SLT, salvage liver transplantation; PLTW, primary liver transplantation for HCC within Milan criteria; PLTB, primary liver transplantation for HCC beyond Milan criteria; TACE, transcatheter arterial chemoembolization.

All the participants received whole liver graft from deceased donors. Different transplant techniques were performed, including 16 cases of classic OLT, 303 cases of modified piggyback technique introduced by YM Wu [4] and 20 cases of classic piggyback. The immunosuppressive regimens used included double regimen (steroid and Tacrolimus or Cyclosporine (CsA)) and triple regimen (steroid, Tacrolimus or CsA, and Mycophenolate mofetil (MMF)). MMF was used in patients with a low serum Tacrolimus concentration even under a relatively high dose intake, and in those patients with hyperglycemia or renal impairment during the early period post-transplantation. When MMF was given, Tacrolimus was maintained in a lower tough level. Liver function and blood concentration of immunosuppressants were monitored according to the protocols in our center. Interleukin-2 receptor monoclonal antibody (Basiliximab) induction was adopted in patients with high-risk factors, such patients with age >60-year old, hypoalbuminemia, hepatorenal syndrome and a model for end-stage liver disease (MELD) score over 30. The interleukin-2 monoclonal antibody was administered intraoperatively and on day 4 post-transplantation, respectively. A dose of 500 mg steroid was administered during operation. When induction therapy was used, Tacrolimus or CsA was used from day 4 post-transplantation, and then was adjusted according to plasma concentration. Prior to the study, the protocol, which was in accordance with the ethical guidelines of the 1975 Helsinki Declaration, was approved by the institutional ethics committee of the First Affiliated Hospital of Sun Yat-sen University. Written, informed consent was obtained from all subjects.

### Statistical analysis

All statistical analysis was performed using the Statistical Package for Social Science 13.0 (SPSS, version 13.0; Chicago, IL). Continuous variables were tested for normal distribution and expressed as mean ± standard deviation (SD) or median (range) as appropriate. Categorical variables were compared by Pearson chi-squared test and continuous variables were compared by Student's t-test. Univariate survival curves were estimated using the Kaplan-Meier method and compared by the log-rank test. Risk factors for tumor recurrence were evaluated by a Cox Proportional Hazards model. For all analyses, *P* values<0.05 were considered statistically significant.

## Results

### Implementation of SLT

Thirty-six patients, including 29 males and 7 females, received SLT after radical HR due to intrahepatic recurrence. Sixteen patients received primary right hemihepatectomy, 10 left hemihepatectomy and the others irregular hepatic segmentectomy pre-transplantation. Before HR, 22 patients had single tumor nodule, 12 had 2 or 3 nodules, and only 2 had >3 tumor nodules. In all patients, the tumors were located within a liver lobe without macrovascular invasion. The post-operative pathologic studies showed poorly differentiated HCC in 24 cases and well differentiated HCC in the other 16 cases. The median interval between initial HR and SLT was 35 months (1–63 months). Among the 36 patients, 15 had received radiofrequency ablation or ethanol injection pre-transplantation, 3 patients received transcatheter arterial chemoembolization (TACE).

### Operative parameters and postoperative complications

The operative parameters and post-operative complications between the two groups of patients were described in Table 2. The intraoperative blood loss (1560±670 ml versus 1180±910 ml, *P*<0.05) and transfusion volume (1060±780 ml versus 820±910 ml, *P*<0.05) were larger in the SLT group than in PLTW group. The operation time was longer in the SLT versus PLTW group (340±77 min versus 302±81 min, *P*<0.05). These indicated that SLT would increase the operation difficulties. However, the postoperative recovery and intraoperative complications between the two groups were not significantly different (*P*>0.05).

**Table 2:** Operative parameters and postoperative complications.

	SLT (*n* = 36)	PLTW (*n* = 147)	*t* value or *χ* ^2^ value	*P* value
Donor liver cold ischemic time (h)	8.1±2.5	7.4±2.8	1.37	0.127
Anhepatic time (min)	39.6±5.2	38.3±6.9	1.06	0.268
Operative time (min)	340±77	302±81	2.54	0.024*
Application of arterial jump grafts	3	2	5.29	0.021
Roux-n-Y	4	3	6.47	0.011
Intraoperative bleeding volume (ml)	1560±670	1180±910	2.35	0.028*
Intraoperative transfusion volume (ml)	1060±780	820±910	2.02	0.043*
Postoperative ICU time (h)	34±12	29±16	1.76	0.078
Primary graft nonfunction	0	0	–	–
Delayed graft function	1	4	<0.001	0.985
Intra-abdominal bleeding	0	4	1.001	0.317
Infections	2	14	0.571	0.450
Renal failure	1	3	0.073	0.786
Acute rejection	2	15	0.742	0.389
Biliary complications	2	14	0.571	0.450
Vascular complications	0	3	0.747	0.387
Recurrence of hepatitis	0	2	0.495	0.482

Abbreviation: SLT, salvage liver transplantation; PLTW, primary liver transplantation for HCC within Milan criteria; ICU, intensive care unit.

### Patient survival

There were 11 deaths in the SLT group, including 1 perioperative death due to severe infection. In PLTW group, there were 36 deaths, including 3 perioperative deaths (1 died from renal failure, 1 from severe infection and 1 from hepatic artery thrombosis). Survival curves generated by the Kaplan-Meier method are shown in Figure 1A. Log-Rank test showed that the patient survival was not significantly different between the two groups (*χ* ^2^ = 0.926, *P* = 0.336).

**Figure 1:** (A) shows the cumulative survival rate between SLT group and PLTW group, a Log-Rank test showed *P* = 0.336. (B) shows the cumulative survival rate between SLT group and PLTB group, a Log-Rank test showed *P* = 0.041. Abbreviation: SLT salvage liver transplantation, PLTW primary liver transplantation within Milan criteria, PLTB primary liver transplantation beyond Milan criteria.

And in those patients undergoing primary OLT for HCC beyond Milan criteria, there were 75 deaths including 7 perioperative deaths (3 from severe infection, 2 from renal failure, 1 from GVHD and 1 from biliary ischemia). Compared with this group of patients, patients in SLT group achieved longer survival (*P*<0.05) (Figure 1B).

### Tumor recurrence and risk factors

By December 2010, all the patients were follow-up 25–83 months. The median follow-up time of SLT group was 61 months. Five patients of the SLT group experienced recurrences during follow-up, with the mean recurrence time of 28.2±15.1 months. Two patients had metastases in the lung, and the other 3 in the liver graft, bone and brain, respectively. While in the PLTW group, the median follow-up time was 62 months, 15 patients experienced recurrences in 30.4±11.8 months, which were also found in lungs (8 cases), liver grafts (5 cases) and bone (2 cases). The recurrence time (*P*>0.05) and recurrence rate (13.9% versus 10.2%, *χ* ^2^ = 0.403, *P*>0.05) were comparable between the two groups. The tumor recurrence profiles of the patients in the two groups are shown in Table 3. The cumulative recurrence rate curves are shown in Figure 2A.

**Figure 2:** (A) shows the cumulative recurrence rate between SLT group and PLTW group, a Log-Rank test showed *P* = 0.525. (B) shows the cumulative recurrence rate between SLT group and PLTB group, a Log-Rank test showed *P* = 0.006. Abbreviation: SLT salvage liver transplantation, PLTW primary liver transplantation within Milan criteria, PLTB primary liver transplantation beyond Milan criteria.

**Table 3:** Survival and tumor recurrence rate.

Group	Cases	Follow-up (month)	Recurrence		Overall survival rate (%)			Tumor-free survival rate (%)		
			Rate	time (month)	1 yr	3 yrs	5 yrs	1 yrs	3 yrs	5 yrs
SLT	36	58.7±20.7	5/36	28.2±15.1	97.2	80.6	69.4	97.1	87.9	74.2
PLTW	147	64.2±18.1	15/147	30.4±11.8	98.0	86.4	75.5	97.9	89.9	80.3
PLTB	156	57.2±33.1	63/156	22.5±14.9	96.2	64.7	48.7	88.5	53.2	33.6
*P* value		0.065	<0.001	<0.001	0.657	<0.001	<0.001	0.002	<0.001	<0.001

Abbreviation: SLT, salvage liver transplantation; PLTW, primary liver transplantation for HCC within Milan criteria; PLTB, primary liver transplantation for HCC beyond Milan criteria.

In 156 patients who received primary OLT for HCC beyond Milan criteria, 63 (40.3%) patients experienced recurrence in 16.5±10.9 months. The recurrence rate was higher in this group of patients compared with SLT group (*χ* ^2^ = 8.977, *P* = 0.003). The cumulative recurrence rate curves are shown in Figure 2B.

A Cox Proportional Hazards model was made to evaluate the risks factors for tumor recurrence in all of the patients here, the result showed that vascular invasion, including macrovascular and microvascular invasion, as well as AFP level >400 IU/L were risk factors for tumor recurrence after LT, as showed in Table 4.

**Table 4:** Risk factors for Overall survival of liver transplantation by Multivariate Analysis.

Items	n	Mean±SD (months)	Univariate analysis	Multivariate analysis
**Age (yr)**			0.192	
<47	169	63.21±2.23		
≥47	170	59.23±3.41		
**Gender (M/F)**			0.241	
Male	251	57.34±2.16		
Female	78	59.54±3.31		
**HBV infeciont**			0.105	
Present	328	58.94±2.16		
Absent	11	62.54±5.31		
**HCV infection**			0.143	
Present	22	59.24±2.16		
Absent	317	61.54±3.31		
**ALT**			0.267	
**<135**	169	63.52±2.34		
≥**135**	170	58.12±3.64		
**MELD score**			0.228	
<18	169	66.21±4.43		
≥18	170	62.03±5.22		
**Liver cirrhosis**			0.312	
**Present**	271	55.34±2.16		
**Absent**	68	59.54±3.31		
**Nodules numbers**			0.109	
≤3	227	65.52±1.54		
>3	62	59.12±2.75		
**AFP levels**			0.001	0.031^a^
<400	66	73.66±2.09		
≥400	273	62.09±1.64		
**Macrovascular invasion**			<0.001	<0.001^b^
Present	37	40.28±4.16		
Absent	302	67.22±2.35		
**Microvascular invasion**			<0.001	0.009^c^
Present	71	46.56±3.46		
Absent	268	69.31±3.45		
**Pathologic characteristics**			0.092	
Poor differentiated	106	62.34±1.46		
Well differentiated	233	59.86±3.17		
**Pre-transplant treatment**			0.185	
Present	164	62.54±3.46		
Absent	175	59.91±4.32		

a Relative risk:1.91, 95% CI: 1.04–3.02.

b Relative risk:3.33, 95% CI: 1.77–6.24.

c Relative risk:2.93, 95% CI: 1.31–6.11. Cox Proportional Hazards model showed that vascular invasion, including macrovascular and microvascular invasion, as well as AFP level >400 IU/L were risk factors for tumor recurrence after OLT.

## Discussion

HCC is one of the most common malignant tumors in China, with the incidence rate up to 80 per million populations. More than 80% patients had simultaneous liver cirrhosis, which leads to an actual rate of resection less than 30%, while the 5 year recurrence rate after resection reached above 70% [3], [5], [6]. Theoretically, OLT was the most effective treatment for HCC patients, which not only achieves radical tumor resection, but also deals with the frequently concurrent end stage liver diseases. In China mainland, nearly half of liver transplant recipients were patients with HCC [7]. However, considering the severe organ shortage, high cost and perioperative risk of this procedure, as well as constraint in concept, HR remains to be the mainstay treatment for patients with resectable early HCC. Although OLT can yield a higher tumor-free survival than HR in early HCC patients with Child A stage liver function, the 5-year survival rate had no significant difference between the two procedures [8]. The reasons might be as follows: (1) the perioperative mortality of liver transplant is higher than that of HR; (2) the survival rate of liver transplant recipients declines because of rejection, recurrence of hepatitis, side effects of immunosuppressants and transplant-related complications; (3) re-excision, radiofrequency ablation and OLT can be applied for recurrence after HR, which prolong patient survival time; (4) due to organ shortage, 15%∼33% of patients lost the opportunities of transplantation because of tumor progression [7], [9], [10].

However, SLT remained a life-saving treatment for patients with intrahepatic recurrence or liver function deterioration after primary HR [2], [10], [11]. In some cases, surgical resection can be taken as an initial treatment so as to control tumor progression when patients are on the waiting list. Transplantation can be implemented as soon as donor liver is available [12]. Previous studies have documented that 80% of patients suffered from intrahepatic recurrence after HR, and about 52% of the recurrent patients are still transplantable [13], [14], [15]. Whether the patients can receive SLT depends on the tumor factors, age of patients, the time waiting for a donor liver, and the patients' willingness.

The surgical difficulty in SLT increases due to peritoneal adhesions caused by previous upper abdominal surgery. The adhesions usually lie between the cut surface and the omentum and/or the intestine. In addition, some recipients may have vigorous portal collaterals, which might lead to massive intraoperative bleeding. The dissection of the liver hilum might be another technical difficulty in SLT, especially when hilar dissection has been done extensively during previous hepatectomy. Several such cases were included in our study, we used the iliac artery from the same donor as a bridge and the celiac trunk of the graft was anastomosed to the recipients' abdominal aorta via the bridge. A Roux-en-Y hepaticojejunostomy was utilized for biliary reconstruction. Although some studies have shown that SLT does not increase the difficulty of surgery [13], [16], [17], the SLT group did have longer operative time, more introperative blood loss and transfusion volume in our study. The interval between initial LR and SLT may be a factor related to the operative difficulty since the severity of adhesion is associated with this interval. However, the increased difficulty neither increases the post-operative complications, nor negatively affects the short and long term prognosis. There was one patient received SLT just 1 month after resection, the later was performed in another hospital. This patient had liver cirrhosis and a tumor with 5 cm in diameter locating at the right lobe, while two susceptive small nodules in S4 was also noted, which was regarded as cirrhotic nodules by the doctors. During the first operation, the cirrhosis was more severe than what had been expected before the operation, right lobectomy was performed. Importantly, a PET-CT scanning one month after the resection revealed that the two nodules in S4 were HCC nodules. Therefore, LT was suggested immediately after the PET-CT scanning. This patient seems more likely had remnant cancer, and he had tumor recurrence about 24 months after transplantation.

Nowadays, the treatment for liver cancer develops rapidly. There are a variety of interventional therapy that can be chosen for recurrence, including radiofrequency ablation, ethanol injection, and TACE. Besides, some studies [14] have shown that SLT has no obvious advantage over the treatment strategies mentioned above. However, most studies still support that transplantation is the most effective treatment for HCC. In this study, we observe that the Milan criteria are still eligible for the 36 patients at the time of recurrence. And the 5-year overall survival rate and disease-free survival rate are not lower than those undergoing primary OLT.

In conclusion, in comparison with primary OLT, although SLT would increase the operation difficulties, it provides a good option for patients with HCC recurrence after curative resection. Identification of recurrent patients who would gain favorable outcomes from SLT will help decision-making among multiple choices of treatment.
